# Deep-Learning-Based Color Doppler Ultrasound Image Feature in the Diagnosis of Elderly Patients with Chronic Heart Failure Complicated with Sarcopenia

**DOI:** 10.1155/2021/2603842

**Published:** 2021-07-29

**Authors:** Peng Bian, Xiyu Zhang, Ruihong Liu, Huijie Li, Qingqing Zhang, Baoling Dai

**Affiliations:** ^1^Department of Statistics and Medical Record Management, Provincial Hospital Affiliated to Shandong First Medical University, Jinan 250021, Shandong, China; ^2^Medical Office, Liaocheng Hospital of Traditional Chinese Medicine of Shandong Province, Liaocheng 252000, Shandong, China

## Abstract

The neural network algorithm of deep learning was applied to optimize and improve color Doppler ultrasound images, which was used for the research on elderly patients with chronic heart failure (CHF) complicated with sarcopenia, so as to analyze the effect of the deep-learning-based color Doppler ultrasound image on the diagnosis of CHF. 259 patients were selected randomly in this study, who were admitted to hospital from October 2017 to March 2020 and were diagnosed with sarcopenia. Then, all of them underwent cardiac ultrasound examination and were divided into two groups according to whether deep learning technology was used for image processing or not. A group of routine unprocessed images was set as the control group, and the images processed by deep learning were set as the experimental group. The results of color Doppler images before and after processing were analyzed and compared; that is, the processed images of the experimental group were clearer and had higher resolution than the unprocessed images of the control group, with the peak signal-to-noise ratio (PSNR) = 20 and structural similarity index measure (SSIM) = 0.09; the similarity between the final diagnosis results and the examination results of the experimental group (93.5%) was higher than that of the control group (87.0%), and the comparison was statistically significant (*P* < 0.05); among all the patients diagnosed with sarcopenia, 88.9% were also eventually diagnosed with CHF and only a small part of them were diagnosed with other diseases, with statistical significance (*P* < 0.05). In conclusion, deep learning technology had certain application value in processing color Doppler ultrasound images. Although there was no obvious difference between the color Doppler ultrasound images before and after processing, they could all make a better diagnosis. Moreover, the research results showed the correlation between CHF and sarcopenia.

## 1. Introduction

Cardiovascular and cerebrovascular diseases are high-morbidity diseases in the elderly population. With the aging of the population in China, the occurrence and mortality of cardiovascular and cerebrovascular diseases are gradually increasing, especially in the aspect of heart. Chronic heart failure (CHF) will appear in the late stage of heart disease development [1]. According to the statistics, the probability of suffering from CHF is between 1.3% and 1.8% in our population at the present stage and 30% to 50% of the CHF patients eventually die [2]. Sarcopenia, also known as age-related sarcopenia, is a complication of developing CHF, which mainly refers to an age-related degenerative syndrome in which the content of human skeletal muscle gradually decreases with the increase of age, as well as the strength and function of muscle gradually deteriorates [3]. The incidence of sarcopenia varies by region and race, but it is a general trend that increases with age, so it can also be called a progressive geriatric syndrome [4]. Studies have shown that grip strength, muscle strength of quadriceps femoris, 6-minute walking distance, reduced left ventricular ejection fraction, and high oxygen consumption will appear due to low exercise peak when CHF patients are complicated with sarcopenia [5]. Moreover, it is proposed that this complication will not only reduce the quality of life of the patients but also increase the probability of death of the patients through the analysis of patients with CHF complicated with sarcopenia [3].

Cardiac color Doppler ultrasound is a major examination method in diagnosing CHF disease, which is now the only imaging method that can display circulation situation in the internal structure of the heart and organs, and the method has simple operation, causes no wound, and can be repeated [6]. When patients with CHF are examined, the cardiac image structure is comprehensively and intuitively displayed, thereby providing a more favorable and reliable basis for doctors' diagnosis [7].

Deep learning is a kind of artificial intelligence technology that has developed very rapidly in recent years. The neural network system of deep learning has made great progress in image classification and examination. Furthermore, this technology is also widely applied in the medical field. Intelligent medical care, which is a combination of deep learning artificial intelligence and the medical industry, has become a research hotspot [8]. It also solves two major problems for the medical industry: the first one is the imbalance between the amount of imaging data and the amount of clinical imaging data, and the second one is the imbalance between the level of imaging doctors and the allocation of resources [9]. Deep learning methods have been fully and reasonably utilized in image processing and analysis in the medical field. In particular, the deep convolutional network model can more effectively learn image features from a large number of samples, avoid the complex feature extraction process in traditional image classification algorithms, and realize end-to-end classification and detection [10].

In this study, deep learning convolutional neural network technology was combined with color Doppler ultrasound images, which was used for the diagnosis of CHF to analyze the correlation between CHF and sarcopenia.

## 2. Methods

### 2.1. Research Objects

A total of 259 patients were randomly selected in this study, who were diagnosed as sarcopenia and admitted to hospital from October 2017 to March 2021, including 119 males and 140 females. They were 60 to 76 years old, with an average age of 69.5 ± 3.5 years. All patients underwent cardiac ultrasound examinations, who were rolled into two groups according to whether deep learning technology was used for image processing or not. A group of routine unprocessed images was set as the control group, and the images processed by deep learning were set as the experimental group. This study was approved by the Medical Ethics Committee, and all the patients participating in the study signed the informed consent forms.

The criteria for inclusion were defined to include patients who were over 50 years of age, were diagnosed as sarcopenia based on the diagnostic criteria proposed by the Asian Working Group for Sarcopenia (AWGS) [11] (Table 1), and were able to undergo a complete color ultrasound examination, whose color ultrasound images were well preserved.

The criteria for exclusion were defined to include patients who had skeletal disease or motor obstruction disease, had previous history of fracture, suffered from diabetes, thyroid, and parathyroid gland and other endocrine system diseases, had diseases of the digestive system and renal insufficiency that affected skeletal muscle metabolism, suffered from malignant tumors and connective tissue diseases, and took calcium, hormone drugs, and antitumor drugs within 1 year, with female ovarian lesions.

### 2.2. Research Methods

#### 2.2.1. Diagnostic Methods of Chronic Heart Failure

For the diagnosis of CHF, the method of combining the clinical manifestations with the results of other auxiliary examinations was adopted to make the combined diagnosis, as shown in Figure 1.

#### 2.2.2. Convolution Neural Network Algorithm Model

In this study, a convolutional neural network algorithm-based color Doppler ultrasound image model would be established according to the pixel resolution and the performance of stable deep neural network. Then, it would be trained and applied in this study.

The convolution layer was set as the layer *q*, so the feature graph of the input color ultrasound image at the layer *q* − 1 could be expressed as follows:

(1) $$\begin{array}{c} W\left(q,p\right)=\sum_{e=1}^{E}Y^{\left(q,p,e\right)}\;⊗\;Z^{\left(q-1,e\right)}+l^{\left(q,p\right)}. \end{array}$$

In addition, *W*^(*q*, *p*, *e*)^ represented the convolution kernel, *l*^(*q*, *p*)^ stood for the bias, and *e* meant the number of feature graphs.

In this study, the commonly used and high-rate ReLu was used as the activation function, which is shown in equation (2), and the corresponding derivative function expression is presented in equation (3). However, due to the excessive data gradient passing through the ReLu neuron, once the data were updated, the neuron would not be able to activate any data again, so it was improved into equation (3). It was a self-gated activation function, which could be called swish.

(2) $$\begin{array}{c} f\left(x\right)=\max\left(0,x\right), \end{array}$$

(3) $$\begin{array}{c} f^{\prime }\left(x\right)=\left\{\begin{array}{cc} x, & x>0,\\ 0, & x\leq 0, \end{array}\right) \end{array}$$

(4) $$\begin{array}{c} F_{1}\left(x\right)=\left(R_{1}*X+L_{1}\right)\times \frac{Y}{Y+u^{-\alpha \left(R_{1}*X+L_{1}\right)}}. \end{array}$$

In equation (4), *R*_1_ stands for the convolution kernel, *i* × *f*_1_ × *f*_1_ expresses the size, *i* indicates the number of channels of the input graph, *L*_1_ represents the offset vector, *∗* means the convolution operation, and *α* stands for the parameter that could be trained.

In this model, the first layer was mainly for the operation of extracting the feature map of the original color ultrasound image, and the second layer to the *q* − 2 layer was the nonlinear mapping process of the extracted feature map, which could be expressed by the following equation:

(5) $$\begin{array}{c} F_{2}\left(x\right)=\left(R_{2}*X+L_{2}\right)\times \frac{Y}{Y+u^{-\alpha \left(R_{2}*X+L_{2}\right)}}. \end{array}$$

The reconstruction process of the image could be expressed as equation (6), where *R*_3_ represents the mean filter and *L*_3_ expresses the offset of dimension *i*.

(6) $$\begin{array}{c} F_{3}\left(x\right)=R_{3}*F_{2}\left(X\right)+L_{3}. \end{array}$$

The convolutional neural network algorithm needed to be reconstructed according to the error, and the parameter error in the propagation process was constantly corrected. If the current propagation was *q*, the output parameter of the layer was *x*^*q*^, and the weight and bias could be expressed by *R*^*q*^ and *L*^*q*^ in turn, as shown in the following equations:

(7) $$\begin{array}{c} x^{q}=f\left(p^{q}\right), \end{array}$$

(8) $$\begin{array}{c} \left(p^{q}\right)=R^{q}x^{q-1}+l^{q}. \end{array}$$

The expression of loss function was as shown in the following equation:

(9) $$\begin{array}{c} \text{Loss}\left(s,s^{\prime }\right)=\frac{1}{n}\sum_{j=1}^{n}{\left(s_{j},s_{j}^{\prime }\right)}^{2}. \end{array}$$

The method of reducing the gradient was adopted to minimize the sum of squares of errors, and the specific algorithm is shown in the following equations:

(10) $$\begin{array}{c} R_{j}=R_{j}-\beta \frac{\chi }{\chi R_{j}}M\left(R,l\right), \end{array}$$

(11) $$\begin{array}{c} R_{j}=R_{jk}-\beta \frac{1}{z}\sum_{j=1}^{z}\left[V_{r,l}\left(x^{j}\right)-s^{j}\right]x^{j}. \end{array}$$

Among them, *β* represents the weight, *χ* represents the volume number, and *s* refers to the loss data.

For the semisupervised learning algorithm aiming at the inherent noise and uncertainty in ultrasonic images, its calculation method was displayed as follows, but the derivation process was omitted:

(12) $$\begin{array}{c} L_{\text{label}}=-B\left[\ln\;g\left(y\;|\;x\right)\right]=-ly+\text{LSE}\left(l\right), \end{array}$$

(13) $$\begin{array}{c} L_{\text{unlabel}}=-E\left[\ln\left(1-g\left(H+1\right)\;|\;x\right)\right]=-\text{LSE}\left(l\right)+\text{sofplus}\left(\text{LSE}\left(l\right)\right), \end{array}$$

(14) $$\begin{array}{c} L_{\text{fake}}=-E\left[\ln\;g\left(H+1\;|\;x\right)\right]=\text{softplus}\left(\text{LSE}\left(l\right)\right), \end{array}$$

(15) $$\begin{array}{c} L_{D}=L_{\text{label}}+\frac{v\left(L_{\text{unlabel}}+L_{\text{fake}}\right)}{2}. \end{array}$$

In equations (12)–(15), *H* stands for the classifier and *H* + 1 means the output graph of the discriminator. The whole system included real data with labels, noise data without labels, and generated data, and the corresponding probabilities were *L*_label_, *L*_unlabel_, and *L*_fake_, respectively.

Figure 2 shows the comparison of the cardiac color ultrasound images before and after processing and optimization by this algorithm.

#### 2.2.3. Evaluation Criteria for the Algorithm Effect

In order to evaluate the effect achieved by the abovementioned algorithm model, the peak signal-to-noise ratio (PSNR) and structural similarity index measure (SSIM) were applied in this study. Besides, the smaller the value of PSNR, the smaller the degree of image distortion. However, the closer the SSIM value was to 1, the more similar the processed image would be to the original. The specific algorithm of PSNR is shown in equations (16) and (17), where *K* expresses the image height, *H* means the image width, and *n* stands for the bit value of each pixel.

(16) $$\begin{array}{c} \text{MSE}=\frac{1}{K\times L}\sum_{i=1}^{K}\sum_{j=1}^{H}{\left(X\left(i,j\right)-Y\left(i,j\right)\right)}^{2}, \end{array}$$

(17) $$\begin{array}{c} P=10\;\log_{10}\left(\frac{{\left(2^{n}-1\right)}^{2}}{\text{MSE}}\right). \end{array}$$

SSIM could be calculated as in equation (18), where *α*_*x*_ indicates the average value of *x*, *α*_*y*_ means the average value of *y*, *β*_*x*_^2^ represents the variance of *x*, *β*_*y*_^2^ stands for the variance of *y*, and *β*_*xy*_ expresses the covariance of *x* and *y*.

(18) $$\begin{array}{c} \text{SSIM}\left(x,y\right)=\frac{\left(2\alpha_{x}\alpha_{y}+e_{1}\right)\left(2\beta_{xy}+e_{2}\right)}{\left(\alpha_{x}^{2}+\alpha_{y}^{2}+e_{1}\right)\left(\beta_{x}^{2}+\beta_{y}^{2}+e_{2}\right)}. \end{array}$$

### 2.3. Observation Indicators

The left atrial diameter (LAD), left ventricular ejection fraction (LVEF), and left ventricular end-diastolic diameter (LVDD) of the two groups were observed and recorded by using a color Doppler ultrasound, so as to evaluate and compare the positive rates of LAD, LVEF, and LCDD in the two groups. Positive criteria for diagnosis of CHF by using the cardiac ultrasound [12]: ① LAD > 30 mm was positive; ② LVDD > 55 mm in male and >50 mm in female were positive; and ③ LVEF < 50% was positive.

The detection results of the two groups were compared, the number of sarcopenia patients diagnosed with CHF was contrasted, and the clinical manifestations and other auxiliary examinations were combined to confirm the diagnosis, so as to analyze the accuracy of the cardiac ultrasound examination.

### 2.4. Statistical Methods

SPSS 23.0 statistical software was used for data processing, in which measurement data were expressed as (*x* ± *s*), and the two independent samples *t*-test was used for comparison between groups. Count data were represented by [*n* (%)], and the *χ*^2^ test was used for comparison between groups. In addition, *P* < 0.05 indicated that the difference was statistically substantial.

## 3. Results

### 3.1. Comparison on Cardiac Color Ultrasound Images of Patients with Chronic Heart Failure and Other Heart Diseases from Two Groups

The cardiac color ultrasound images of patients from the two groups were observed, clearly showing that the processed images of the experimental group were clearer than the untreated images of the control group, which also had higher resolution. Therefore, it indicated that the deep learning convolutional neural network algorithm had a certain effect on optimization for color ultrasound images, and the specific comparison is shown in Figures 3 and 4. In addition, PSNR and SSIM were adopted to evaluate the effect of processing, achieving good results (PSNR = 20 and SSIM = 0.09).

### 3.2. Comparison of LVEF, LCDD, and LAD Results between the Two Groups

By statistical analysis of the diagnostic results of LVEF, LCDD, and LAD in the two groups of cardiac color ultrasound of all patients (Table 2), it was found that the indicators of LVEF, LCDD, and LAD of the control group were lower than the indicators of the experimental group, and the comparison was statistically significant (*P* < 0.05), as shown in Figure 5.

### 3.3. Statistical Comparison on the Positive Rates of LVEF, LCDD, and LAD Results from Cardiac Color Ultrasound Diagnosis between the Two Groups

There was statistical analysis on the positive rates of diagnostic results of LVEF, LCDD, and LAD in the two groups of heart color ultrasound of all patients (Table 3).  Figure 6 reveals that the positive rates of LVEF, LCDD, and LAD of the experimental group were higher than the rates of the control group, and the comparison was statistically significant (*P* < 0.05).

### 3.4. Comparison on the Results of CHF Patients Diagnosed in the Two Groups and the Final Confirmed Results

Table 4 shows the comparison of the number of patients diagnosed with CHF by using the cardiac color ultrasound and the final diagnosis combined with other clinical examinations. The study results suggested that the similarity between the final diagnosis results and the examination results of the experimental group was 93.5%, while the similarity between the results and the control group was 87.0%. Thus, the similarity between the experimental group and the control group was higher, and the comparison was statistically significant (*P* < 0.05). Among all the patients diagnosed with sarcopenia in this study, 88.9% were also finally diagnosed with CHF, and only a small part suffered from other diseases, which showed statistical significance (*P* < 0.05). In contrast, 77.2% of the patients from the control group and 83% from the experimental group had the combination of the two diseases. There was statistical significance in comparing the probability of patients with CHF among the three groups (*P* < 0.05), as shown in Figure 7.

## 4. Discussion

In today's medical field, the application of medical imaging technology in the screening, diagnosis and treatment, and evaluation of clinical diseases has become more and more extensive, and it is a very critical examination method [13]. Since the diagnosis and evaluation of image maps in the past was mainly carried out by excellent doctors and they had the uneven experience level, the results of the review were very different, and it was also highly subjective [14]. Therefore, as the deep learning artificial intelligence technology research has achieved excellent results, the technology has been extensively used in all aspects of the medical field, especially in the improvement and promotion of medical imaging technology, and has achieved good research results, showing good results in clinical examination and diagnosis [15]. At this stage, the medical imaging technology system and medical image processing and analysis are the most typical application scenarios of medical technology based on deep learning methods, and significant results have been achieved.

In this study, the neural network algorithm of deep learning was adopted to optimize and improve the color Doppler ultrasound images, which was applied in the diagnosis of CHF complicated with sarcopenia. The comparison of images before and after processing showed that the algorithm model had certain effect on image improvement, not only for color Doppler ultrasound image processing but also for other commonly used imaging techniques such as CT and MRI. Voets et al. [16] reported on the diagnosis of diabetic retinopathy in the *Journal of the American Medical Association*. It was proved that the end-to-end deep learning model could be directly applied to medical image processing, and the diagnostic results obtained were very similar with experts, which were even better than the diagnosis made by experts. Varghese et al. [17] combined imaging with machine learning (ML) to cross examine the accuracy of multiple ML algorithms for the detection of clinically significant PCa (csPCa). The results showed that the second kernel-based support vector machine (SVM) had the best accuracy, up to 92%. Zhang et al. [18] applied MSCTA three-dimensional reconstruction technology in the treatment of colorectal cancer. By comparing the consistency of the MSCTA three-dimensional reconstruction with the actual surgical plan, they found that the kappa consistency test between the two was *k* = 0.769, which proved MSCTA three-dimensional reconstruction had a good effect in guiding the treatment of colorectal cancer under laparoscopy.

In this study, CHF patients complicated with sarcopenia accounted for a large part of the total number of patients, which fully reflected that there was a certain connection between the two. Besides, the correlation between CHF and sarcopenia was extensively investigated. Some experts conducted a statistical study on 200 CHF patients with an average age of 70.8 ± 8.3 years, and the results showed that the incidence of CHF with sarcopenia was 19.5% [19]. A large number of studies have shown that 68% of patients with CHF are complicated with muscle fiber atrophy, the body mass of elderly patients with CHF is decreased, and the decreased exercise tolerance may be related to skeletal muscle fiber and skeletal muscle mass loss [20]. By exploring and analyzing CHF patients complicated with sarcopenia, foreign research experts have found recently that there is a certain correlation between skeletal muscle decline and pathological changes such as coronary atherosclerosis in elderly people and have proposed that sarcopenia may also have a reliable influence on the disease development of CHF [21]. Those mentioned above were similar to the results of this study, and there was a close correlation between CHF and the occurrence of sarcopenia.

## 5. Conclusions

In this study, the deep learning neural network algorithm is used to optimize and improve the color Doppler ultrasound image for the diagnosis of CHF complicated with myopenia. It is found that the processed image of the experimental group is clearer and has higher resolution than the unprocessed image of the control group. The final diagnosis result is more similar to the experimental group, which also indicates the correlation between CHF and myopenia. However, due to the limitation of the research scope, this study lacks a certain representativeness. However, the overall results show that the application of deep learning artificial intelligence in the field of imaging is still very promising.

## Figures and Tables

**Figure 1:** Diagnostic criteria for CHF.

**Figure 2:** Comparison on cardiac color ultrasound images before and after optimization by convolutional neural network algorithm.

**Figure 3:** Comparison on cardiac color ultrasound images of CHF patients between the two groups. (a) Control group; (b) experimental group.

**Figure 4:** Comparison on cardiac color ultrasound images between the two groups of patients with other heart diseases. (a) Control group; (b) experimental group.

**Figure 5:** Comparison on the results of LVEF, LCDD, and LAD diagnosed by using a cardiac color ultrasound between the two groups.

**Figure 6:** Comparison on positive rates of LVEF, LCDD, and LAD diagnosed by using a color Doppler ultrasound between the two groups.

**Figure 7:** Comparison on the probability of patients with CHF in the three groups.

**Table 1:** Diagnostic criteria for AWGS sarcopenia.

	Evaluation content	Gender	Criteria
One	The mass of skeletal muscle measured by the dual energy X-ray absorption method; calculation of the ratio of the mass to the height square	Male	<7.0 kg/m^2^
		Female	<5.4 kg/m^2^

Two	Grip strength	Male	<26 kg
		Female	<18 kg
	Walking speed	6-minute walking speed	<0.8 m/s

*Note*. Patients who met any of these criteria could be diagnosed with sarcopenia.

**Table 2:** Statistical results of LVEF, LCDD, and LAD diagnosed by using a cardiac ultrasound in the two groups.

Indicators	Group	
	Control group	Experimental group
LVEF (%)	54.05 ± 4.79	60.09 ± 4.34
LCDD (mm)	51.35 ± 3.97	56.05 ± 3.09
LAD (mm)	33.45 ± 4.01	40.05 ± 4.12

**Table 3:** Statistical results of positive rates of cardiac ultrasound in LVEF, LCDD, and LAD in the two groups.

Indicators	Positive rate (*n* %)	
	Control group	Experimental group
LVEF (%)	56	65
LCDD (mm)	59	69
LAD (mm)	57	66

**Table 4:** Comparison on the results of CHF patients diagnosed from the two groups and the final diagnosis results.

Symptom	Group		
	Control group	Experimental group	The final diagnosis results
CHF	200	215	230
Other diseases	59	44	29
CHF proportion	77.4%	83.1%	88.9%

## Data Availability

The data used to support the findings of this study are available from the corresponding author upon request.
